This article has been retracted.

# Exploring Evaluation of Enterprise Economic Benefits Using Big Data

**DOI:** 10.1155/2022/1103561

**Published:** 2022-06-28

**Authors:** Xiaoqian Liu, Yujia Li

**Affiliations:** ^1^Green Innovation Industrial Institute, School of Economics and Management, Chengdu Technological University, Chengdu 610000, China; ^2^School of Business College, Changchun Guanghua University, Changchun 130000, China

## Abstract

The purpose is to improve Chinese enterprises' economic benefit evaluation system based on big data and promote sustainable enterprise production. This paper studies the power supply enterprises-oriented Evaluation Index System (EIS) under the big data environment. Firstly, it expounds on the construction theory of the enterprise economic benefit model. Secondly, the comprehensive Grey Model (GM) based on improved weight and the power consumption prediction model based on Least Mean Square (LMS) neural network (NN) algorithm are introduced. Finally, the comprehensive GM model based on improved weight is used to evaluate the economic benefits of power supply enterprises. The power consumption prediction model based on the LMS-NN algorithm is used to predict the sustainable development of power supply enterprises. The results show that the profitability and solvency of joint-stock power companies are about 90 and 100, respectively, and the social contribution of state-owned power supply enterprises is the strongest. Lastly, it is predicted that the region will have 134.8 billion kWh of electricity and about 137.2 billion kWh of power consumption in 2020. The growth model and trend are consistent, but there are some errors in the specific power consumption data. Therefore, the audit method based on big data has a good evaluation effect on the economic benefits of enterprises. For example, the profits of private and joint-stock power supply enterprises are relatively high. In contrast, state-owned power supply enterprises have outstanding social contribution ability. The big data method is used to predict the power consumption in some areas, and the predicted value is consistent with the actual value. This study provides a reference for the follow-up economic benefit evaluation and sustainable development of enterprises.

## 1. Introduction

Enterprises are the main vitality of national and social-economic development, and the economic benefits of enterprises are the foundation of their existence and development because all the behaviors and management activities of an enterprise are carried out based on economic benefits. Electric power enterprises are an important part of the national economy and energy supply, as well as the basis for the national economy and national financial revenue [1]. The rise and fall of electric power enterprises will fundamentally affect the national social economy and energy security, which means that the economic benefits of their enterprises will also affect the national fiscal revenue and the sustainable development of energy. Because of their particularity and importance to the country, power supply enterprises may be different from other industries, and even monopolistic behaviors may occur. Although the relevant departments of the national government have taken many methods and measures, little effect has been achieved. The biggest problem of power enterprises is that there is no competition. In other words, some power supply enterprises or companies have no sense of competition in the whole industry market, which leads to low enthusiasm within the enterprises, which makes the environment of power supply enterprises complicated and then directly affects the economic effect of enterprises [2]. Therefore, an Evaluation Index System (EIS) should be established for enterprise economic benefits. This is of great help for analyzing the profitability of power supply enterprises and solving their existing problems.

With the rapid development of information technology, Internet technology based on big data has been integrated into various industries in people's lives and has a very broad prospect in energy utilization fields, such as power engineering. Due to the rapid development of the electric power industry, traditional data processing methods have been unable to deal with related applications faster and more accurately, so the use of big data method has become the best data processing method for modern enterprises, including power supply enterprises. Big data is not just cloud computing that expands the amount of simple data. Compared with traditional statistical methods, big data can quickly find and process data. When operating on interconnected data, it also considers the relationship between the data. It can find problems and reduce risks, to achieve the required work effect [3]. Big data also has a good application effect in the evaluation of the economic benefits of enterprises. Particularly, data information sharing and intercommunication can be realized by applying the big data audit record method to the economic benefit review and evaluation, establishing an economic benefit EIS for electric power enterprises, and evaluating and storing the economic benefit data of each power supply area or unit. This is conducive to the analysis of benefit evaluation data, thus discovering and solving relevant problems improving the economic benefits of the enterprise, and reducing the risk of unfavorable factors. Nations are carrying out prototype research on the Internet of Energy (IoE) like Germany and Japan with small-scale pilot applications. In 2008, Germany selected six pilot areas based on smart grid to carry out the four-year *E*-Energy technology innovation promotion plan and the national natural science foundation project “Future Renewable Power Energy Transmission and Management System.” Foreign scholar Rokita-Poskart (2017) established an enterprise economic benefit EIS using financial and nonfinancial indicators, such as financial leverage ratio, activity ratio, profit, and loss ratio [4]. Afterward, the economic benefits of some enterprises are evaluated through similar technology priority methods and a fuzzy Analytic Hierarchy Process (AHP). IoE technology has also attracted widespread attention in China. China's State Grid has also proposed and promoted the global IoE strategy. Domestic scholars Liu et al. evaluated the comprehensive benefits of selected listed companies using the factor analysis method [5]. The results obtained by the model analysis were consistent with the development performance of listed companies.

To sum up, China's enterprise economic benefit EIS is not perfect, and relevant research is scarce. At present, enterprise financial data cannot be well audited and counted. Particularly, some power supply enterprises have problems, such as imperfect economic benefit audit, incomplete financial data, information exchange, untimely revenue, and expenditure. Therefore, this paper researches domestic power supply enterprises using Big Data Technology (BDT) and improves their economic benefit EIS. It realizes the sustainable development of enterprise production capacity. It aims to provide a reference for the subsequent economic benefit evaluation and sustainable development of enterprises. The innovation of this paper is that the comprehensive Gray Model (GM) based on improved weight is used to evaluate the economic benefits of power supply enterprises. The power consumption prediction model based on Least Mean Square (LMS) NN algorithm is used to predict the sustainable development of power supply enterprises.

## 2. Methods

### 2.1. Enterprise Economic Benefit Model Construction Theory Elaboration

#### 2.1.1. Enterprise Economic Benefit Evaluation

Enterprise economic benefit is also called financial-economic benefit evaluation, which is essentially an evaluation of enterprise financial benefit from the perspective of financial revenue forecast and enterprise management. Among them, the profitability and debt repayment ability of an enterprise are two very important indicators to evaluate the economic benefits of an enterprise, which can be used to judge the economic benefits of an enterprise, such as its operating status, financial revenue, and sustainable development feasibility [6].

#### 2.1.2. The Big Data Audit Method

The big data audit is an emerging data processing technology based on big data in the Internet environment. Big data audit can carry out network-based cloud computing for simple and complex data, use the network or database to search and obtain the required data, show the relationship and association of these data, and show the data changes and dynamic trends by algorithm-built models [7]. The big data audit method can determine the processing order of data audit, thus realizing the static and dynamic simulation analysis of data and the data control and monitoring from the field to the remote. The economic benefit EIS of electric power enterprises is established by applying the big data audit method to the economic benefit of enterprises. The evaluation and storage of the economic benefit data of each power supply area or unit and the realization of data information sharing and communication are conducive to the development of the benefit EIS of enterprises.

#### 2.1.3. Financial Performance Indicators

The traditional economic evaluation of power generation projects mainly focuses on financial benefit analysis. The main idea is to discount the project's cash inflow and cash outflow at an appropriate discount rate and calculate the Financial Net Present Value (FNPV). Then, FNPV is used to judge the project's profitability by comparing it with the number 0. Under the background of a low-carbon economy (LCE), power generation enterprises may face many uncertain profit-making factors. This calculation method does not fully reflect the real benefits of power generation projects. The calculation results may affect the Decision-Making (DM) of power generation enterprises on relevant projects. In particular, carbon emissions and carbon tax and other factors can be introduced into the economic benefit evaluation of power generation projects from the perspective of the enterprise. Doing so can value some hidden benefits of low-carbon power generation projects and then correctly evaluate the economic benefits of power generation projects. The financial benefit indicators of enterprises are usually evaluated through Financial Net Present Value (FNPV), Internal Rate of Return (IRR), Dynamic Investment Payback Period (PP), and ROI (Return of Investment), including dynamic and static indicators [8], thus realizing project financial decisions. Here, the low-carbon benefit indicator is used to evaluate the economic benefit of power supply enterprises. In this way, the financial revenue and profitability of power supply enterprises in the low-carbon economy can be analyzed and expressed intuitively and systematically during the calculation period to ensure the sustainable development of economic benefits of enterprises. The selection of low-carbon financial benefit indicators is shown in Figure 1.

#### 2.1.4. NN

The NN is a kind of nonlinear network structure based on the structure and function of the animal or human brain, which can be divided into two kinds: biological NN and artificial neural networks (ANN). In machine learning and net-related neighborhood, the animal NN is generally used [9]. NN is composed of interconnected neural units that can be used to predict and analyze large amounts of input data or some relatively complex unknown approximate functions. Because there is a nonlinear relationship between thinking, logic, and analysis in the brain and intelligence, the nonlinear relationship is also common in nature. According to the complexity of the target object or research thing, the NN can realize the process of hiding or expressing the data by changing the interrelation between the network nodes, namely, the weight value. Moreover, the NN has the characteristic of self-learning. The NN can use the training and deep learning process to readjust the structure, adapt to the needs of different data information processing and storage, and better express the relationship between input and output information data [10].

#### 2.1.5. Weight Determination Method

Weight determination methods can be divided into subjective weight method, objective weight method, and subjective and objective weight method. The subjective weighting method has the advantage of the relative concentration of experience and opinions and can modify the data in continuous feedback according to the subjective consciousness or importance of each indicator to obtain the required results. Indicator comparison method, two-way assignment method, and binomial coefficient method are commonly used subjective weighting methods. The objective weighting method is a statistical method that uses the information of indicators to determine the decision matrix. The weight of the matrix is obtained by objective operation, and the entropy method is commonly used. The objective weighting method combines the subjective weighting method and the objective weighting method. A certain weight coefficient is allocated so that the determined weight can reflect subjective and objective information.

### 2.2. Construction of Enterprise Economic Benefit Evaluation Model

#### 2.2.1. Determination of the Weight of Indicators

The established quantitative indicators can intuitively calculate data. In order to make the evaluation more objective, the entropy method and Analytic Hierarchy Process (AHP) are used to determine the objective weight and the subjective weight, respectively. Then, the objective and subjective weights are combined based on a specific coefficient to obtain the combination weight coefficient of the evaluation index.

First, the economic evaluation indicators of enterprises are selected, and the weights of each indicator can be determined by subjective and objective weighting methods, as shown in Figure 2.

The subjective and objective weighting method distributes certain weight coefficients so that the determined weight can reflect the subjective and objective information [11].

Here, subjective and objective weighting methods are used to determine the quantitative indicator of enterprise economic benefit evaluation. The objective weight of economic benefit is determined by the entropy method. AHP is used to determine the subjective weight of economic benefits. Then, the combination coefficient is used to evaluate the results obtained by the two methods and then the combined weight coefficient of the evaluation indicator is obtained.

#### 2.2.2. The Entropy Value Method

Standardization of data: due to different dimensions of different indicators, the initial data are standardized and comparatively analyzed [12]. The standardized expression reads

(1) $$\begin{array}{c} y_{ij}=\frac{x_{ij}}{\sum_{i=1}^{n}x_{ij}}. \end{array}$$

In (1), *y*_*ij*_ refers to the contribution degree of the ITH scheme in the JTH indicator attribute. *x*_*ij*_ refers to the indicator of the ITH scheme in the JTH indicator attribute.

The calculation of the entropy of the JTH indicator, *e*_*j*_, reads

(2) $$\begin{array}{c} e_{j}=-k\sum_{i=1}^{m}y_{ij}\ln\;y_{ij}, \end{array}$$

where *e*_*j*_ refers to the total contribution of all schemes to the second indicator and *k* refers to a constant. When all schemes in the indicator attribute are close to the same, the total contribution of all schemes to the third indicator will be close to 1. When the contribution is close to the same, it means that the indicator attribute has no role in the decision, so when the target attribute is not considered, the value of the target attribute can be determined as 0 [13].

(3) $$\begin{array}{c} g_{j}=1-e_{j}, \end{array}$$

where *g*_*j*_ is the differential coefficient of an indicator. The larger the value of *g*_*j*_, the more the attention paid to the role of the indicator.

(4) $$\begin{array}{c} w_{j}^{1}=\frac{g_{j}}{\sum_{i=1}^{n}g_{j}}, \end{array}$$

where *w*_*j*_^1^ determines the weight coefficient.

#### 2.2.3. Comprehensive Evaluation Model of Gray Correlation Method

During the evaluation matrix determination, the fuzzy AHP has strong subjectivity and uncertainty [14]. Here, the gray correlation method is used to determine the value of the economic benefit evaluation matrix. The correlation coefficient between the reference sequence and comparison sequence is used to judge the difference between different power supply enterprises. The comparison sequence of indicators for each scheme reads

(5) $$\begin{array}{c} x\left(j\right)=\left\{x\left(1\right),x\left(2\right),x\left(3\right)\ldots x\left(n\right)\right\}. \end{array}$$

*i*=1,2,3,…, *n* is the number of schemes.

The indicators are preprocessed. The indicators adopted here include power generation capacity *A*1, profitability *A*2, debt repayment capacity *A*3, financial maintenance capacity *A*4, and social contribution capacity *A*5.

Parameter sequence selection: parameter series is the evaluation standard for each economic benefit. The parameter sequence corresponds to the evaluation indicator and is the set of the best quality; that is, the optimal indicator is selected. For example, when the indicator indicates profitability, the maximum value should be calculated and selected to reflect the profitability of the power supply enterprise. The expression of the reference sequence reads

(6) $$\begin{array}{c} x_{1}\left(j\right)=x_{1}\left(1\right),x_{1}\left(2\right),x_{1}\left(3\right),\ldots ,x\left(n\right). \end{array}$$

In (6), *i*=1,2,3,…, *n* represents the number of schemes.

Further, the indicators are nondimensionalized [15]. The dimensions of evaluation indicators differ. Before the evaluation, the dimensionless indicator information can be unified to reduce the interference from random factors.

The correlation coefficient is calculated. The correlation coefficient is calculated from the comparison sequence and the reference sequence through the matrix.

### 2.3. Prediction of Power Consumption Sustainability Based on the NN Algorithm

#### 2.3.1. Neuron Model

Linear purelin function is used in the neuron model [16]. The neuron model is shown in Figure 3.

#### 2.3.2. NN Structure

A NN consists of many neurons, and each neuron can have an output. As shown in Figure 4, their relationship is shown in the following equation:

(7) $$\begin{array}{c} y=\text{purelin}\left(w*p+b\right). \end{array}$$

In (7), *p* refers to the input one-dimensional vector, *b* is the deviation matrix, *y* represents the output matrix, and *w* is the weight matrix. Purelin function is used for calculation.

#### 2.3.3. Windrow-Hoff Learns the Rules

W-H learning rule (Windrow-Hoff) is a judgment standard for NN convergence based on the Least Mean Square (LMS) algorithm proposed by Windrow and Hoff. The group of W-H learning rules is used to modify the weight vector. The process of the perceptron is simplified by error-correcting learning rules to make it simpler [17]. The calculation process is shown in Figure 5.

The function of the linear NN is to process the mean-variance of the resulting error so that it can be reduced to the lowest value. That is, the actual output is determined at an optimal value, and the lowest result error can be obtained using the following equation:

(8) $$\begin{array}{c} e\left(n\right)=d\left(n\right)-x\left(n\right)*w\left(n\right). \end{array}$$

In (5), *d*(*n*) refers to the expected output, *x*(*n*) and *w*(*n*) represent the actual output, respectively, and *e*(*n*) denotes the error between the expected output and the actual output.

#### 2.3.4. LMS Learning Algorithm Training Process

First is the variables and parameters' setting. Specifically, *W*(*n*) and *X*(*n*) are set as the weight vector and the input vector, respectively, and their expressions read

(9) $$\begin{array}{c} X\left(n\right)={\left[1,x_{1\left(n\right)},x_{2\left(n\right)},x_{3\left(n\right)},x_{4\left(n\right)},\ldots ,x_{m\left(n\right)}\right]}^{T}, \end{array}$$

(10) $$\begin{array}{c} W\left(n\right)={\left[w_{1\left(n\right)},w_{2\left(n\right)},w_{3\left(n\right)},w_{4\left(n\right)},\ldots ,w_{m\left(n\right)},\right]}^{T}, \end{array}$$

where *X*(*n*) is the input vector, namely, the training sample, *W*(*n*) represents the weight vector, *m* and *n* are the numbers of input vectors, and *T* is the number of iterations.

A relatively small random nonzero value is assigned to *W*_*j*_(0) to initialize the weight vector. For a set of input samples *X*(*n*) and the corresponding expected output *d*, *e* (*n*) is calculated, and iteration is computed [18]. The specific expression reads

(11) $$\begin{array}{c} W\left(n+1\right)=W\left(n\right)+\eta X^{T}\left(n\right)*e\left(n\right). \end{array}$$

In (11), *e* (*n*) represents the error between the expected output and the actual output, and *η* is the calculation coefficient.

Then, the results are judged; if the results meet the convergence conditions, the algorithm can be finished. If the convergence condition is not met, the *n* value needs to be increased by 1 and returned to the third step [19]. The required condition is that the error of the calculation result is less than the specified value *ε*; that is, the error value between the expected output and the actual output is less than *ε*. The weight change is very small, so the absolute value of the change in the weight vector is less than *ε*. Additionally, the number of iterations should be set, namely, the number of limits. When the number of iterations reaches the specified number or the highest iteration value, the algorithm will end. In this way, the algorithm calculation can be prevented from entering an infinite loop, resulting in no result or incorrect result [20].

The experimental data are Beijing's population and economic data from 2000 to 2020 from the 3E sustainable development platform according to the values of multiple factors affecting power consumption. At the same time, some resource websites are reviewed, such as the Beijing Statistical Yearbook and the National Bureau of Statistics, to collect Beijing's social power consumption data from 2000 to 2020. Through regression analysis, historical data can be obtained.

## 3. Results

### 3.1. Analysis of Influencing Factors of Economic Benefit Evaluation of Power Supply Enterprises Based on Big Data

This experiment takes private, state-owned, and joint-stock power supply enterprises as the research object. The economic benefit EIS of power supply enterprises reported here mainly decomposes the economic benefit audit objectives, such as economy, efficiency, and effectiveness. It uses the balanced scorecard method in the four dimensions of finance, customers, internal business process, learning, and growth. There are two-level indicators and three-level indicators under the four dimensions. The three-level indicators adopt combined qualitative and quantitative methods to refine and set different evaluation indicators. Five indicators are set for evaluation, including power generation capacity *A*_1_, profitability *A*_2_, debt repayment capacity *A*_3_, financial maintenance capacity *A*_4_, and social contribution capacity *A*_5_.

Table 1 and Figure 6 show that the economic benefit evaluation ability of private and joint-stock electric power companies is higher than that of state-owned electric power enterprises on the whole. The difference between a private electric power company and a joint-stock electric power company is not very big, the data size of different indicators is not the same, and they both have their specific advantages. For example, the profitability and solvency of joint-stock power companies are around 90 and 100, respectively. And in terms of social contribution, it is much better than private power enterprises. The power generation capacity and sustainable development capacity of private power supply enterprises are the highest among the three power supply enterprises. Moreover, the profitability of private enterprises is similar to that of stock power enterprises, but their social contribution is relatively small, which needs to be improved. Overall, private power supply enterprises are worse than joint-stock power supply enterprises. The analysis shows that state-owned power supply enterprises have the worst economic benefit evaluation. Hence, state-owned power supply enterprises have poor economic benefits, and there are also big problems in profitability and solvency. The evaluation indicators are relatively low, and even negative economic growth may occur. But state-owned power supply enterprises have great advantages over private enterprises and joint-stock enterprises in terms of social contribution ability, because state-owned power supply enterprises themselves have certain policies to benefit the people [21], and they can be maintained despite poor economic benefits.

### 3.2. Prediction Results of Sustainable Development Based on Big Data Method

The electricity consumption situation of some areas from 2000 to 2016 is input into the prediction model [22], and the predicted value is shown in Figure 7. Figure 7 indicates that the electricity consumption in this area increases steadily at a certain rate. In 2020, there are 134.8 billion kilowatt-hours of electricity in the area, which is relatively high. When electricity consumption is around 137.2 billion KWH, the growth pattern and trend are relatively consistent. But there are some errors in the specific data of electricity consumption.

Table 2 demonstrates that the relative error of the prediction model based on the LMS-NN algorithm is smaller than that of the regression model and gray prediction model. Although the trend of electricity consumption predicted by the three models is the same, the growth rate is different. The actual value of electricity in the area is also different. The prediction effect of the LMS-NN is much better than that of the regression model and GM, and it is more accurate in some specific electricity data. For example, from 2011 to 2015, certain measures are taken to control population growth in the region due to the implementation of the sustainable development strategy. Therefore, the growth rate of electricity consumption during this period has declined and the trend has slowed down. The regression model and GM have a large prediction error for this phenomenon and do not show this trend well. The fitting effect of the LMS-NN is very good, and the prediction model shows this trend. This is because the LMS algorithm can obtain a relatively high convergence speed when the number of weights of the NN is small, reduce iterations, improve prediction accuracy, and minimize the mean error variance. That is, the actual output is determined at an optimal value, and the equation can be used to obtain the lowest error. In conclusion, the power consumption prediction model based on the LMS-NN algorithm can predict power consumption sustainability.

Overall, the comprehensive GM based on improved weight is used to evaluate the economic benefits of power supply enterprises. It is concluded that the audit method based on big data has a good effect on the evaluation of the economic benefits of enterprises. According to the economic benefit evaluation of power supply enterprises under different indicators, private power supply enterprises and joint-stock power supply enterprises have high profitability and solvency. The ability of state-owned power supply enterprises in the social contribution is more prominent than other enterprises. The prediction model based on the LMS-NN algorithm is used to study the sustainable development of power consumption of power supply enterprises. The big data method is used to predict power consumption in some areas. The trend of the predicted value is consistent with the actual value, and the prediction of power consumption sustainability is realized.

## 4. Conclusion

This paper mainly studies power supply enterprises-oriented economic benefit EIS in the big data environment. Firstly, it expounds on the construction theory of the enterprise economic benefit model and puts forward a big data audit method for the power supply enterprises-oriented economic benefit EIS. Then, the comprehensive GM model based on improved weight is used to evaluate the economic benefits of power supply enterprises. Besides, the sustainable development of power consumption of power supply enterprises is studied using the prediction model based on the LMS-NN algorithm. The results show that the audit method based on big data has a good effect on evaluating enterprise economic benefits. According to different indicators, private and joint-stock power supply enterprises have higher profitability and solvency than state-owned enterprises. The state-owned power supply enterprises are prominent in social contribution ability. According to the prediction of power consumption in some areas, it is concluded that the power consumption of the whole region will be 134.8 billion kWh in 2020, which is relatively high. The growth model and trend are relatively consistent when the power consumption is about 137.2 billion kWh. However, there are some errors in the specific data of power consumption. The trend of the predicted value is consistent with the actual value, and the prediction of power consumption sustainability is realized. Although the economic benefits of enterprises are evaluated, and the sustainability of electricity consumption is predicted by combining the big data method, the collected enterprise data and model parameters still have errors. There is a certain gap between the predicted data and the actual data, which needs further research and improvement. Future research will study the NN, Support Vector Machine (SVM), and other models and combine them with sufficient experimental data. Based on this, it can make a reasonable prediction for the next 50 or even 100 years. More scientific-technical means promote the improvement and development of enterprise economic benefit EIS and contribute to the sustainable development of energy in China.

## Figures and Tables

**Figure 1:** Financial benefit evaluation indicators.

**Figure 2:** Quantitative framework of enterprise economic benefit evaluation based on big data and subjective and objective weighting method.

**Figure 3:** Neuron model.

**Figure 4:** Network structure diagram.

**Figure 5:** W-H learning rule calculation process.

**Figure 6:** Evaluation of operation economic benefit of different power supply enterprises.

**Figure 7:** Comparison of the actual and predicted value of electricity consumption (only predicted value after 2021).

**Table 1:** Indicators of different power supply enterprises.

Type of power supply enterprise	Total indicator	*A*_1_	*A*_2_	*A*_3_	*A*_4_	*A*_5_
Private	0.6604	1.0004	0.9581	0.5200	0.9876	0.4830
State-owned	0.2413	0.0832	0.000	0.0000	0.2563	0.5508
Joint-stock	0.6802	0.2365	0.9732	1.0036	0.6980	0.5071

**Table 2:** Comparison of prediction models based on different algorithms (*A* is regression model, *B* represents GM, and *C* denotes LMS-NN model).

Time	Electricity consumption per billion kilowatt-hours	*A* the relative error (%)	*B* the relative error (%)	*C* the relative error (%)
2011	660.01	3.90	−4.82	−0.70
2012	690.70	0.45	−2.25	1.05
2013	740.20	1.90	−3.35	0.60
2014	809.90	2.70	−6.40	0.20
2015	823.21	−2.16	−2.09	0.52
2016	874.28	−1.09	−2.40	0.50
2017	918.11	−1.30	−0.88	4.08
2018	938.01	−3.60	2.50	0.15
2019	960.80	−6.70	6.95	−1.38
2020	1028.27	−8.90	6.01	0.16

## Data Availability

The simulation experiment data used to support the findings of this study are available from the corresponding author upon request.
